# Deep Learning-Based Computed Tomography Imaging to Diagnose the Lung Nodule and Treatment Effect of Radiofrequency Ablation

**DOI:** 10.1155/2021/6556266

**Published:** 2021-10-20

**Authors:** Xixi Guo, Yuze Li, Chunjie Yang, Yanjiang Hu, Yun Zhou, Zhenhua Wang, Liguo Zhang, Hongjun Hu, Yuemin Wu

**Affiliations:** ^1^Department 2 of Thoracic Oncology, Xinxiang Central Hospital, Xinxiang 453000, Henan, China; ^2^Disinfection and Supply Center, Liyang People's Hospital, Liyang 213300, Jiangsu, China; ^3^Department of Thoracic Surgery, Liyang People's Hospital, Liyang 213300, Jiangsu, China

## Abstract

This study aimed to detect and diagnose the lung nodules as early as possible to effectively treat them, thereby reducing the burden on the medical system and patients. A lung computed tomography (CT) image segmentation algorithm was constructed based on the deep learning convolutional neural network (CNN). The clinical data of 69 patients with lung nodules diagnosed by needle biopsy and pathological comprehensive diagnosis at hospital were collected for specific analysis. The CT image segmentation algorithm was used to distinguish the nature and volume of lung nodules and compared with other computer aided design (CAD) software (Philips ISP). 69 patients with lung nodules were treated by radiofrequency ablation (RFA). The results showed that the diagnostic sensitivity of the CT image segmentation algorithm based on the CNN was obviously higher than that of the Philips ISP for solid nodules <5 mm (63 cases vs. 33 cases) (*P* < 0.05); it was the same result for the subsolid nodule <5 mm (33 case vs. 5 cases) (*P* < 0.05) that was slightly higher for solid and subsolid nodules with a diameter of 5–10 mm (37 cases vs. 28 cases) (*P* < 0.05). In addition, the CNN algorithm can reach all detection for calcified nodules and pleural nodules (7 cases; 5 cases), and the diagnostic sensitivities were much better than those of Philips ISP (2 cases; 3 cases) (*P* < 0.05). Patients with pulmonary nodules treated by RFA were in good postoperative condition, with a half-year survival rate of 100% and a one-year survival rate of 72.4%. Therefore, it could be concluded that the CT image segmentation algorithm based on the CNN could effectively detect and diagnose the lung nodules early, and the RFA could effectively treat the lung nodules.

## 1. Introduction

There are about 600,000 new lung cancer patients worldwide every year. As a malignant tumor with the highest morbidity rate, lung cancer has brought severe challenges to people's life safety [1]. The number of deaths of lung cancer patients in China is close to one-fifth of cancer deaths. Early detection and diagnosis and early treatment of lung cancer are the key to effectively reduce their mortality [2]. In the early stage of lung cancer, the main symptom is the appearance of nodules with a diameter of no more than 3 cm in the patient's lungs. Early diagnosis and treatment of lung nodules can help improve the quality of life and survival rate of patients. However, due to the small diameter of lung nodules, how to accurately locate the lung nodules has become a key issue [3].

In the earliest days, people mainly diagnosed pulmonary nodules by imaging methods [4], mainly including X-ray diagnosis and computed tomography (CT) diagnosis. X-ray diagnosis uses different relative densities of different parts of the human body, and the absorption rate of X-rays is not all similar. Based on this feature, X-rays are transmitted through the human body to produce images. However, due to technical reasons, X-rays cause the lesions or lung nodules to be slightly larger than the actual situation, which is easy to mislead the patient's diagnosis and treatment. With the advancement of science and technology, CT imaging came out. CT uses computer technology to divide the human body from the horizontal level by pixels. It can detect the relative densities of different parts by changing the position of the X-ray and the orientation of the detector receiving the signal according to the strength displayed on the detector, further displaying the human body scan image [5]. Compared with X-ray examination, CT examination can detect lung nodules with a smaller volume, which helps medical staff to correctly diagnose lung nodules and adopt reasonable treatment methods [6].

How to accurately locate and detect lung nodules so as to detect, diagnose, and treat lung nodules as early as possible is worthy of our attention [7, 8]. Lung nodule detection algorithms generally mainly consist of image analysis and pattern recognition. The original CT image includes lung parenchyma, fat, and other internal tissues and organs of the human body, bones, and background images. The focus of this study was lung nodules, which mainly distributed in the lung parenchyma [9, 10]. In recent years, the newly proposed deep learning has the function of automatically finding relative features because each image has a different shape, and the errors caused by human factors can be adjusted through deep learning. At present, as a deep learning structure based on visual perception, the convolutional neural network (CNN) has received a lot of attention from researchers because they are closer to biological neural networks [11]. In this study, a CNN method was proposed to diagnose and discover the lung nodules early. Compared with other method structures, the utilization of features is higher, and the amount of calculation is less. It can effectively reduce the complexity of the model and reduce the amount of operation while ensuring the accuracy. In addition, there is no need for complex preprocessing of images, and it is suitable for application development in the context of big data. Using the CNN can help medical workers treat patients with pulmonary nodules earlier and better and reduce the burden on the medical system and patients [12].

The latest development of radiofrequency ablation (RFA) [13] can treat patients with lung nodules who have lost surgical treatment opportunities or are not suitable for surgical treatment to a certain extent. It can directly kill tumor cells in the patient while avoiding the impact on the patient's lung function. Compared with methods such as surgery and chemotherapy, patients need less cost and shorter hospital stay, which is worthy of clinical promotion [14]. The content of this study is the application of CT images based on deep learning of the CNN in the diagnosis of lung nodules and the application of RFA treatment of lung nodules under the guidance of CT. It was expected that deep learning can be more effectively and accurately applied in the early diagnosis of lung nodules, providing a more detailed reference basis for medical workers to select treatment options.

## 2. Materials and Methods

### 2.1. Research Objects and Grouping

The clinical data of 69 pulmonary nodule patients diagnosed by needle biopsy and pathological comprehensive diagnosis in hospital from January 2020 to January 2021 were collected for analysis, including 35 males and 34 females, with an average age of 53 ± 7.62 and the median age of 63 years old. The maximum diameter of pulmonary nodules ranged from 10 mm to 30 mm, and the average size was 21 mm. A total of 69 needle biopsy was performed, and there were 69 lesions in total. The process had been approved by the ethics committee of hospital, and all the subjects included in the study had signed the agreements.

The inclusion criteria were defined as follows: patients whose CT examination showed no significant changes in lung nodules within half a year; patients older than 18 years old; patients with normal blood coagulation without treatment; patients with complete imaging data, complete surgical records, and pathological results before surgery; and patients with reasonable examinations, clinical treatments, and theoretical analysis.

The exclusion criteria were determined as follows: patients whose image quality did not meet the standard to affect the observation; patients without other major diseases in addition to lung nodules, such as impaired heart, liver, and kidney functions, blood system diseases, malignant tumors, and mental diseases; and patients with coagulation dysfunction detected before the surgery.

### 2.2. CT Image Segmentation Algorithm Based on the CNN

The CNN improves the current existing CT image detection algorithm. As a kind of the deep learning method, it effectively improves the learning efficiency of artificial intelligence and also ensures the stability of the detection rate.  Figure 1 shows the algorithm flowchart of the CNN.

According to the previous algorithm flow, the area of lung parenchyma can only occupy a small part of the entire lung CT image, and the lung nodules existing in the lung parenchymal area occupies a smaller area. The CT image of the lung parenchymal region had to be segmented before detection, which was segmented by the method of region growth. Region growth is to group the pixels with similar properties in the CT image into one place and iterate in sequence until the segmentation is completed. The specific steps were as follows. A point in the seed area was selected as the seed point, which was marked as *x*, and the average and standard deviation of the pixel gray level in the seed area were calculated. The seed point was undertaken as the core to check whether the pixel gray value difference of adjacent points was within the allowable error range. If it matched, it would be merged into the seed area; if it did not match, it would be discarded. The merged new point was undertaken as the center to check the neighboring pixels, which was iterated sequentially until the segmentation was completed. The pixel gray average and standard deviation of the seed area were recalculated and reiterated until no more pixels were merged into the segmented area.

Comparison of Figures 2 and 3 shows that the segmented lung parenchyma image was also difficult to identify the difference between blood vessels, bronchus, and lung nodules, so the blood vessels and bronchus were taken as regions of interest, and the lung parenchyma was divided into region of interest (ROI) and air. Then, the lung nodule was marked in the ROI and compared with blood vessels and bronchus to eliminate them. After the features of the ROI were determined, these features had to be classified. The most recent approach was generally used in medicine to classify. It was supposed, there were a type of pattern recognition, which were marked as *w*_1_, *w*_2_,…, *w*_*a*_, and there were *N*_*i*_ for each sample; then, its function was specified as follows.

(1) $$\begin{array}{c} g_{i}\left(x\right)=\text{min}\left\|x-x_{i}^{k}\right\|,\;k=1,2,\ldots ,N_{i}. \end{array}$$

The subscript *i* of *x*_*i*_^*k*^ represents the *w*_*i*_ type, and *k* represents the *k*^th^*N*_*i*_ sample of the *w*_*i*_ type. Cross-information entropy is often used in deep learning for image segmentation. In this study, the small batch stochastic gradient descent was adopted to optimize the obtained CT images. Then, the specific equation for the cross-information entropy loss of CT images is as follows:

(2) $$\begin{array}{c} ℒ=-\frac{1}{N}\underset{i，j，k}{\sum }\left[y_{ijk}^{t}*\text{log}y_{ijk}^{p}+\left(1-y_{ijk}^{t}\right)\mathrm{*log}\left(1-y_{ijk}^{t}\right)\right], \end{array}$$

where *Y*_*ijk*_ represents the probability that the *xyz* axis coordinate (*I*, *j*, *k*) was located in the lung nodule in the obtained three-dimensional CT image, and *N* refers to the sum of all the coordinate points of the detected CT image. Since the diameter of the lung nodules was very small, it only accounted for a very small part of the overall lung CT image. Therefore, the image block of the area was marked by the lung nodules to expand the sample.

It was translated within the radius of the nodule; the CT image was flipped according to the sagittal plane and the coronal plane; and the CT image was rotated every 90° in the cross-section. Then, it was adaptively adjusted according to the cross-information entropy loss function weighted by adaptive pixels. The specific equation was written as follows:

(3) $$\begin{array}{c} w_{ijk}=\left\{\begin{array}{cc} \frac{1}{\sum_{uvw}y_{uvw}^{t}} & y_{ijk}^{t}=1\\ \frac{3}{\sum_{uvw}\left(1-y_{uvw}^{t}\right)} & y_{ijk}^{t}=0 \end{array}\right.,\\ {ℒ}_{\text{adapt}}=-\frac{1}{4}\underset{i}{\sum }\underset{j}{\sum }\underset{k}{\sum }\omega_{ijk}*\left[y_{ijk}^{t}\mathrm{*log}\;y_{ijk}^{p}+\left(1-y_{ijk}^{t}\right)*\log\left(1-y_{ijk}^{p}\right)\right]. \end{array}$$

After the above steps, a CT segmentation algorithm based on the CNN was established, and the lung CT images of patients with pulmonary nodules were segmented for corresponding comparative analysis.

### 2.3. CT Examination and Evaluation Methods

The patients were scanned with GE lightspeed 64-slice spiral CT in the United States. The scanning parameters were given as follows: tube voltage was 120 kV, tube current was 300 mA, pitch was 0.9, layer thickness was 2.5 mm, and matrix was 521 × 521. After the CT scan was performed and the scan results were obtained, two experienced senior associate chief physicians with more than five years of experience were invited to jointly check the obtained CT images blindly, and the participation of subjective factors that may affect the results should be avoided as much as possible. If there was a disagreement between the two physicians, a third expert with the same seniority could further analyze and study the controversial image results. The final result was subject to the consensus of the three people after consultation, which could serve as the gold standard. CT images of the patients were divided into three groups based on the size of the nodules, namely, <5 mm group, 5–10 mm group, and >10 mm group. The nodules were classified into calcified nodules and noncalcified nodules according to their density, and noncalcified nodules were further categorized into solid nodule and subsolid nodule. The nodules in special parts were mainly included in pleural nodules.

Before needle biopsy, the general conditions of the patients were evaluated. Then, the patient was instructed to take a proper position according to the position of the lung nodule in the patient's lungs under the guidance of CT, so that the distance from needle insertion point to the position of the lung nodule should be as short as possible. What needed attention was to avoid the patient's bones, blood vessels, trachea, and other related organs and tissues. Then, the RFA needle was inserted into the lung nodules, and the lung nodules were cut and biopsied first, and then, RFA was used for treatment. The ablation apparatus was turned on, the power was set to 150 W, and the initial temperature was adjusted to 90°C. CT examination was performed on the patient's lungs immediately after treatment to observe the relevant pathophysiological conditions.

### 2.4. Experimental Environment

The hardware platform used in this study were described as follows: the operating system was open source Ubuntu16.04; center processing unit (CPU) was Intel i7-8700k; graphics processing unit (GPU) was NVIDIA 1080 Ti; memory size was 188 G; graphics card was NVIDIA Corporation GK210GL (Tesla K80), and video memory size was 11 G. The software platform was Windows10, Keras/TensorFlow, and Python 3.6.

### 2.5. Diagnostic Criteria

In this study, the sensitivity and accuracy of lung nodule detection were adopted to measure the comprehensive performance of the algorithm proposed. The results of surgical pathological examination were defined as the standard to evaluate the results of the patient's CT diagnosis. The sensitivity and accuracy of the proposed algorithm were compared with those of other CAD software (Philips ISP) in segmentation in the diagnosis of lung nodules. In addition, the difference of the consistency between the two groups and the intraoperative or pathologically confirmed consistency was analyzed.

The calculation methods of precision, sensitivity, and specificity can be expressed as follows:

(4) $$\begin{array}{c} \text{PRE}=\frac{\text{TP}}{\text{TP}+\text{FP}},\\ \text{SEN}=\frac{\text{TP}}{\text{TP}+\text{FN}},\\ \text{SPE}=\frac{\text{TN}}{\text{FP}+\text{TN}}. \end{array}$$

In the above equations, PRE, SEN, and SPE refer to the precision, sensitivity, and specificity, respectively. False negative (FN) refers to a negative sample, which was actually a positive sample. False positive (FP) refers a positive sample which was actually a negative sample. True negative (TN) refers to a negative sample, which was actually a negative sample. True positive (TP) refers to a positive sample, which was actually a positive sample.

### 2.6. Statistical Analysis

The SPSS22.0 software was adopted for statistical analysis. The count data were expressed as the number of cases or percentages, and the chi-square test was used for comparison (the sensitivity and specificity were compared using the paired chi-square test), and the measurement data were expressed as the mean ± standard deviation, with the *t*-test for comparison. The inspection level was *α* = 0.05. When *P* < 0.05, the difference was considered to be statistically significant.

## 3. Results

### 3.1. Comparison on the Segmentation Effects of Algorithms on CT Images

Figure 2 shows the original CT image of a patient with pulmonary nodules, and Figure 3 shows the CT image after region growth segmentation and cropping. It illustrated that the CT images after the region growth segmentation and cropping can highlight the image characteristics of the lungs and show the lesions more clearly, showing a better segmentation effect.

### 3.2. Sensitivities of Two Algorithms in Different Nodules

According to the standard, there were a total of 195 nodules, including 101 subsolid nodules, 82 solid nodules, 7 calcified nodules, and 5 pleural nodules.

As shown in Figure 4, the comparison clearly revealed that in the diameter <5 mm group, the sensitivity of the CNN (63 cases) was significantly better than that of Philips ISP (21 cases) (*P* < 0.05); in the 5–10 mm group, the CNN (15 cases) was slightly better than Philips ISP (14 cases), but the difference between the two was not statistically significant (*P* > 0.05); while in the >10 mm group, there was no difference in detection sensitivity between the two algorithms.

The sensitivities of the two algorithms to subsolid nodule are shown in Figure 5. It revealed that the detection sensitivity of the CNN in the <5 mm group was much better than that of the Philips ISP (33 cases vs. 5 cases) (*P* < 0.05) and that in the 5–10 mm group was obviously better compared with the Philips ISP (37 cases vs. 28 cases) (*P* < 0.05), and it was slightly better than Philips ISP in the >10 mm group, showing no statistically observable difference (16 cases vs. 15 cases) (*P* > 0.05).

The sensitivities of the two algorithms to pleural nodules and calcified nodules are analyzed as shown in Figure 6. The CNN algorithm can detect all pleural nodules (7 cases) and calcified nodules (5 cases), and its detection sensitivity was greatly better in contrast to that of Philips ISP (2 cases and 3 cases) (*P* < 0.05).

### 3.3. RFA under the Guidance of CT Images Based on the CNN

All 69 patients successfully completed the RFA treatment, and the surgical complications are given in Table 1.

The survival rate of 69 patients after RFA is shown in Figure 7. After the first half year, the survival rate was 100%, and the survival rate was 72.4% one year later. It can be considered that the use of RFA for patients with pulmonary nodules under the guidance of CT imaging could effectively improve the survival rate of patients.

### 3.4. Comparison on CT Images before and after RFA

The CT images of a male patient with typical lung nodules before and after RFA were compared. The main clinical manifestations of the patient were fever, cough, and chest tightness. CT examination was performed before surgery (Figure 8), the density of the lung was slightly increased, the bronchi and blood vessels were patchy mostly, and a small number of lobules, so the patient was diagnosed as ground-glass pulmonary nodules. CT examination after RFA treatment (Figure 9) showed that patient's lung nodules disappeared and the density returned to normal, which was close to normal lung CT. It can be considered that RFA had a good effect on the treatment of pulmonary nodules.

## 4. Discussion

With the continuous development of CT technology and the continuous shrinking of the scanning distance, the number of CT images is also increasing. Medical workers are slow to process a large amount of CT data and easily lead to physical and mental fatigue of the workers. Therefore, the computer is used for effective classification, preprocessing, and diagnosis of CT images, showing very important research significance [15]. In this study, a segmentation algorithm based on the CNN was proposed to segment the lung CT images of patients with lung nodules, which improved and optimized the diagnosis of lung nodules in lung CT images, showing relatively high robustness. Therefore, it could be well adapted to the lung CT images obtained by multiple devices. Lung nodules are the presymptoms of lung cancer. How to effectively and accurately diagnose the benign and malignant lung nodules has always been a hotpot that plagues medical workers. In medicine, lung nodules are commonly used, and the shape and size of the nodule and the multiplication rate are used for diagnosis [16]. With the advancement and development of science and technology, CT examination can effectively help medical workers make relevant diagnosis of lung nodules, can more accurately show the location and size of lung nodules, and can detect lung nodules autonomously. If the CT images of the same patient at different times show a significant increase in the volume of the lung nodule, it can be determined that the lung nodule is malignant. The traditional algorithms can effectively identify solid lung nodules in CT images, but they fail to effectively confirm the ground-glass lung nodules at the edge of the lungs and the lung nodules that adhere to the bronchus or blood vessels [17]. The CT image segmentation algorithm based on the CNN proposed in this study could accurately and automatically segment various types of lung nodules, including solitary lung nodules, adhesion lung nodules, and ground-glass lung nodules. Generally speaking, lung nodules appear as bright in the middle and dark on both sides in lung CT images. The segmentation algorithm based on the CNN could ensure that the characteristics of lung parenchyma can be accurately displayed in the subtlest part.

Through experimental comparison, it was found that compared with Philips ISP, the CT segmentation algorithm based on the CNN showed a good diagnostic advantage for solid nodules, subsolid nodules, calcified nodules, and pleural nodules with a diameter of <5 mm; there was a slight advantage in the diagnosis of solid nodule and subsolid nodule with a diameter of 5–10 mm; and there was no obvious difference in diagnosis of the solid nodule and subsolid nodule with a diameter of >10 mm. The analysis of the survival rate of 69 patients after surgery showed that the survival rate of the patients after the first half of the year was 100%, and the survival rate after one year was 72.4%. Such results were better than the results of the study by Lv et al. [18]. CT image guidance of artificial intelligence algorithms has a positive impact on radiofrequency ablation of patients with pulmonary nodules and can effectively improve the survival rate of patients.

## 5. Conclusion

In this study, a CT image segmentation algorithm was established based on the CNN to effectively classify the lung nodules. The results disclosed that the CT image segmentation algorithm proposed could effectively detect and diagnose the pulmonary nodules at an early stage and clearly distinguish their nature and size. In addition, RFA could effectively treat patients with pulmonary nodules and ensure a good survival rate. However, in clinical applications, it was not enough to distinguish only the nature and volume of lung nodules. In some cases, it was necessary to distinguish the benign and malignant lung nodules. In addition to lung disease, other tissues, organs, and bones may also have disease, which require further integration. Moreover, the CT image segmentation algorithm based on the CNN proposed in this study was practical to be applied in the clinic. The results of this study showed some limitations due to the small sample size, so its reliability had to be further expanded in the future. But it was believed that with the continuous advancement of science and technology, medical imaging and computer-related technology will be more perfect for the diagnosis and treatment of lung nodules, which will benefit the masses of people.

## Figures and Tables

**Figure 1:** Flowchart for the CNN algorithm.

**Figure 2:** Original CT images of a patient with pulmonary nodules.

**Figure 3:** CT images after region growth segmentation and cropping.

**Figure 4:** Comparison on sensitivities of two algorithms in solid nodules. ^*∗*^The difference was statistically obvious in contrast to Philips ISP (*P* < 0.05).

**Figure 5:** Comparison on sensitivities of two algorithms in subsolid nodules. ^*∗*^The difference was statistically obvious in contrast to Philips ISP (*P* < 0.05).

**Figure 6:** Comparison on sensitivities of two algorithms in pleural nodules and calcified nodules. ^*∗*^The difference was statistically obvious in contrast to Philips ISP (*P* < 0.05).

**Figure 7:** Number of survived patients after RFA.

**Figure 8:** CT image of a patient with lung nodule.

**Figure 9:** CT image of a patient with lung nodule after RFA.

**Table 1:** Complications after RFA under the guidance of CT image.

	Hemoptysis	Pneumothorax	Total number
Number (cases)	7	13	20
Proportion (%)	10.14	18.84	28.96

## Data Availability

The data used to support the findings of this study are available from the corresponding author upon request.
